This article has been retracted.

# Development of College Students' Resilience Scale

**DOI:** 10.1155/2022/8418279

**Published:** 2022-09-23

**Authors:** Yin Wu

**Affiliations:** Mental Health Education and Consultation Center, Students' Affairs Division, Nanjing University of Finance and Economics, Nanjing 210023, China

## Abstract

In order to explore the dimensions of college students' resilience and compile a measuring tool for contemporary Chinese college students' resilience, semistructured interviews are conducted with 20 college students who have experienced adversity, and the initial dimension of college students' resilience is obtained. Based on the initial dimensions, the project is compiled to form the “College Students' Resilience Scale,” which is tested for 1374 college students, and four dimensions of the scale are obtained through exploratory factor analysis. The college students' resilience scale consists of 26 items with 4 dimensions, namely, “self-efficacy and adaptability,” “positive cognition,” “negative emotion adjustment ability,” and “perceived use of social support.” The self-made college students' resilience scale has good reliability and validity and is an effective measuring tool for college students' resilience.

## 1. Introduction

The American Psychological Association defines resilience as the process of good adaptation when an individual faces life adversity, trauma, tragedy, threat, or other major stressors. Resilience is the process of effectively coordinating, adapting, or managing resources under pressure or trauma. Individuals' inner resources, their life experiences, and environment together promote this adaptability and recover from adversity. In a person's life, the experience of resilience is different. Resilience can be defined by the existence of protective factors or processes that mitigate the relationship between stress and risk.

Based on the definition of trait-oriented resilience, many researchers have compiled resilience evaluation tools. The resilience scale (RS) has 25 items, which consists of two subscales: individual ability, self-acceptance, and life acceptance. Connor-Davidson Resilience Scale (CD-RISC) is a commonly used measurement tool in the study of resilience at home and abroad. The scale consists of 25 items and consists of five subscales: personal ability, tolerance of negative emotions, acceptance of change, control, and mental influence. “Chinese Adult Resilience Scale” contains 30 items, including five dimensions: internal control, coping style focusing on problem solving, optimism, personality tendency to accept and use social support, and acceptability. Outcome-oriented researchers measure resilience indirectly from the positive adaptation results after adversity, and evaluation focuses on the phenomena or results of good adaptation after adversity, such as external behavior, emotional/psychological/mental state.

From the definition of resilience, because the concept of resilience itself has many attributes such as ability, process, and result, the conceptual operation and the reliability and effectiveness of evaluation have become one of the bottlenecks in the study of resilience. Ability orientation, result orientation, and process orientation all reflect the essential attributes of resilience, and there is a certain corresponding relationship between them. For example, ability characteristics will affect the resilience process, and ability and process will affect the result. However, compared with the other two statements, the process theory is more meaningful for intervention. It is important to know what resilience is, but it is urgent for us to know the intervening factors in the development of resilience and give full play to its positive effects.

The rest of this paper is organized as follows: Section 2 discusses related work.  Section 3 is the study selection and assessment of methodological quality. The quality of the studies and meta-analysis are discussed in Section 4.  Section 5 concludes the paper with summary.

## 2. Related Work

Social support was a dimension in most process-oriented resilience scales. Resilience scale for adults (RSA) and adolescent mental resilience scale were widely used in China [1, 2]. Liu et al. pointed out in a meta-analysis that at present, the mainstream research on resilience generally tended to realize that the development of resilience was the product of complex interaction between individuals and social and ecological determinants [3]. Actual social support was the support and help from the outside world that individuals actually received in difficult situations, while perceived social support was the expectation and evaluation of social support and the belief of individuals in possible social support. However, these two components were not clarified in the previous definition of “social support” in resilience. Because the measurement scale of resilience was basically a self-rating scale, the “social support” involved often belonged to the social support of individual subjective experience and comprehension from the actual connotation. An online cross-sectional study recruiting 2,993 participants was conducted in China, from 1 to 10, February 2020. The relationship between risk perception, social support, and mental health was examined using multivariate linear regression analyses [4, 5].

Positive cognition was a dimension emphasized by the evaluation scale including result orientation, ability orientation, and process orientation. Of course, the expressions and emphases used in different scales were different, for example, the resilience scale (RS) contains “Acceptance of Self and Life” dimension. Subjective cognition of unfavorable situation was one of the important factors of resilience [6]. Luthar et al. pointed out that disadvantages depended to a great extent on the subjective perception of the parties [7]. People with strong adaptability were better at or use cognitive reevaluation more frequently. Some of the process neurobiological mechanisms included memory inhibition, memory consolidation, and cognitive control of emotions, which reduced emotional response by reinterpreting the meaning of negative stimuli [8].

The items in the dimension of self-efficacy and adaptability basically came from the originally designed “self-efficacy and value” and “problem solving ability.” After exploratory factor analysis, some items in the original two dimensions converged into this new dimension. Connor-Davidson Resilience Scale contained control or internal control dimensions [9]. With regard to the embodiment of emotional state in resilience, the resilience scale for adolescents (RESA) and the adolescent mental resilience scale included “emotional response” and “emotional control” dimensions [10, 11]. Positive emotions contributed to a healthier cognitive response and reduced the awakening of autonomic nerves. In individuals who remained optimistic in the face of trauma, the median dopamine pathway might be more responsive to rewards and more resistant to stress. Polizzi et al. pointed out that emotion regulation could promote emotion and problem-centered coping, thus promoting the development of resilience [12].

## 3. Qualitative Study on the Structure of College Students' Stress Resistance

This part collects and analyzes the data through semistructured in-depth interviews and adopts grounded theory research paradigm to code and analyze the collected qualitative data step by step. On this basis, it summarizes and analyzes the composition dimensions of college students' resilience.

### 3.1. Interviewees

In this study, 20 college students who have experienced adversity in primary and secondary schools and universities and have basically recovered from adversity are interviewed in four universities in Nanjing and Chengdu by using the method of “purpose sampling.” Among them, there are 10 students from Nanjing University's “Inspirational Star” selection of outstanding players, through understanding the evaluation data of the winners in this evaluation. In addition, through the way of electronic poster recruitment and snowballing, another 10 college students who meet the interview requirements are recruited in other three universities for interviews.

Among the interviewees, there are 9 boys and 11 girls. The main adversities experienced by them involve family problems (such as bereavement, divorce of parents, family conflicts, family financial difficulties, staying experience), interpersonal problems (such as encountering school bullying), learning problems (such as learning pressure, failure in college entrance examination), and environmental adaptation problems at different stages, which are representative in terms of adversity types and predicament intensity. According to the principle of “theoretical saturation,” after interviewing 20 respondents, “theoretical saturation” is basically reached; that is, collecting new data can no longer generate new theoretical insights and reveal new properties of core theoretical categories and then stop interviewing new of respondents.

### 3.2. Interview Process

A semistructured interview outline is designed around personal life course, adversity events, coping resources, reactions under adversity, coping styles, and changes after adversity. The interview mainly includes the following aspects: (1) briefly describe the important events in my life experience, including the peaks and valleys. (2) Describe the two most important setbacks before going to college. Describe the feelings, thoughts, actions and personality characteristics in these two dilemmas, and the influence of family, companions and friends, school environment, and other surrounding social environment on the dilemmas. What changes you have made after getting out of the predicament, and what impact this adversity experience has on coping with the predicament later. (3) Describe the two most important setbacks experienced after going to college. Also describe the related problems involved in part 2 above. Describe the differences and similarities in dealing with setbacks before and after going to college. (4) Describe a successful event in the course of life.

The interview is completed by the researcher himself and three graduate students majoring in psychology.

### 3.3. Coding Analysis of Interview Data

After finishing the verbatim draft of the interview, all the interview data are imported into the qualitative analysis software QRS Nvivo 12.0, which is used as an auxiliary tool for data coding and analysis. The content analysis method of grounded theory is used to analyze the transcribed interview data. Grounded theory analysis paradigm is a qualitative research method, which is proposed by Glaser and Strauss in 1967 and has been widely used in the field of social sciences at present. The grounded theory method adopts the method of establishing theory from bottom to top based on empirical data. Grounded theory pays attention to starting with data, adopts inductive analysis, and carries out three-level coding analysis on data through open coding, relational coding, and core coding.

In this study, a doctoral student and a master student majoring in psychology are invited to co-code the same verbatim interview in the open coding stage. First, three coders encode the first third of the content of the interview separately, and then discuss the results of their respective encoding, trying to form a more consistent encoding idea. After that, the three coders continue to complete the last two-thirds of the content coding and then continue to discuss and communicate the coding inconsistencies to see if they could reach an agreement.

Through three-level coding, there are eight categories of internal and external factors that promote college students' positive and good adaptation and recovery in the process of coping with adversity; that is to say, the preliminary results of college students' resilience dimension include eight dimensions, including: self-efficacy, problem solving ability, goal focus, positive cognition, tolerance and acceptance, negative emotion regulation ability, social communication ability, and social support.

1. Self-efficacy helps individuals keep confidence and hope for themselves and the future in adversity. In the interview, it is reflected in the self-affirmation and self-encouragement of individuals in difficulties and the sense of control in the face of difficulties
2. Problem solving ability enables individuals to effectively deal with problems and crises through various channels. In these interviews, many interviewees talk about the way to face problems and deal with them on a case-by-case basis, instead of avoiding them. At the same time, it can effectively solve the problem by looking for information, self-reflection, adaptation, and adjustment
3. Goal focus means that individuals can continue to insist on not giving up under difficulties and pressures. Interviewees mention that they should persist in working hard in difficult situations, keep their inner requirements and goals, and be responsible for themselves
4. Positive cognition enables individuals to look at the influence of problems and dilemmas positively and comprehensively. In the interview, we have positive expectations for the future, can look at difficulties dialectically and comprehensively, and are willing to accept adjustments
5. Tolerance and acceptance help individuals face reality, accept themselves and others, and keep a stable state of mind in adversity. Respondents talk about the attitude of letting nature take its course and the mentality of self-acceptance and tolerance in unfavorable situations
6. Negative emotion adjustment ability enables individuals to recover from negative emotions caused by adversity or stress events. In the interview, it is reflected in the open-minded attitude, and when negative emotions occur, the emotional state can be adjusted in time by diverting attention and self-combing
7. Social communication ability is the influencing factor that affects individuals to obtain external support. Many interviewees talk about ability to understand others effectively, be good at interacting with others, and develop good interactive relationship with others
8. Social support is the care, understanding, acceptance, and support from the outside world that can get under adversity, which promotes and supports the adaptation and recovery of individuals under difficulties. In the interview, the interviewees say that they have received support

## 4. Preliminary Test of College Students' Resilience Scale

### 4.1. Forming Initial Measurement Table

Starting from these eight dimensions, we start to compile the initial project from two aspects: (1) according to the eight dimensions constructed above, based on the original narration obtained in the interview, compile the scale items, and (2) learn from the related items of the existing mature resilience scale.

First of all, we extract projects reflecting the connotation of contemporary college students' resilience through in-depth interviews and carry out the preparation of initial projects. In-depth interviews are conducted with 20 college students, and the interview contents are changed into verbatim manuscripts, which are extracted and analyzed repeatedly in the form of memos. The classified verbatim manuscripts are extracted and analyzed; that is, the core meaning of respondents' answers is analyzed, and they are itemized, and similar items are merged to extract 40 items. Secondly, this study systematically combs the compilation history of stress resistance evaluation tools, which is convenient for reference and learning relevant experiences.

After the formation of the preliminary measurement form, 767 college students are selected from two universities in Nanjing for preliminary measurement by cluster sampling, by means of centralized notification of class students by counselors, including 399 boys and 368 girls. There are 358 freshmen, 308 sophomores, and 101 juniors. Excluding invalid questionnaires that are obviously not completed seriously, such as choosing the same answer for all questions, and obviously contradicting the results of more than two reverse scoring questions and agreed positive scoring questions, a total of 562 valid questionnaires are received. The valid samples include 251 boys and 311 girls. There are 264 freshmen, 224 sophomores, and 74 juniors.

Item analysis is carried out by discriminant index *D*, *CR*, item total correlation method, and item consistency test.

The total scores of the scale items are sorted from high to low, and the first 27% are high, and the last 27% are low. The discrimination index of items 23, 35, 40, 41, and 56 in the 62 items of the preliminary measurement table is less than or equal to. 2.

Independent sample *T* test is carried out on the scores of high and low groups in each item. It is found that there is no significant difference between high and low groups in 1, 2, 3, 4, 5, 6, 12, 13, 17, 18, 19, 20, 21, 22, 24, 37, 38, 39, 42, 46, 47, 50, 60, and 61.

The sample data for factor analysis needs to meet certain conditions. First of all, the sample size should not be too small and should be more than 5 times of the number of variables. Secondly, variables need to be correlated. If variables are independent of each other, common factors cannot be extracted. It can be examined by Bartlett spherical test. If the test is significant, it is suitable for factor analysis, otherwise it is not suitable. Thirdly, the stronger the partial correlation between variables, the better the effect of factor analysis. The partial correlation degree of variables can be judged by KMO test. *KMO* coefficient is very suitable for factor analysis above.

According to the theory of factor analysis, the factor load value of a project can explain the correlation between the project and the common factor. The greater the load value of a project on a certain public factor, the closer the relationship between the project and the public factor.

Table 1 is the factor structure of college students' resilience scale. It is clearly evident from Table 1 that the discrimination degree of 26 questions is done again, and the discrimination degree of all items is greater than 0.6.

### 4.2. Formal Test and Reliability and Validity Test of College Students' Resilience Scale

In the sampling process, the distribution of samples such as region, grade, and school level should be properly considered. From Nanjing University, Zhejiang University, Nanjing University of Aeronautics and Astronautics, a total of 1,458 college students are selected from 16 schools. 84 invalid questionnaires are eliminated, and 1,374 valid questionnaires are obtained, with an effective rate of 94.24%. There are 538 boys and 836 girls. There are 542 freshmen, 428 sophomores, 275 juniors, and 129 seniors. There are 260 students in science, 343 in engineering, 183 in humanities and social sciences, 413 in economic management, and 175 in other categories.

Table 2 is reliability coefficient of internal consistency of college students' resilience scale. It is clearly evident from Table 2 that the internal consistency coefficient of each factor is between.84 and.94, which has good homogeneity reliability.

Table 3 is test-retest reliability of college students' resilience scale. It is clearly evident from Table 3 that among them, the overall test-retest reliability of the scale is.67, and the test-retest reliability of each dimension is between.42 and.69, and all of them reach the significant level, which shows that the questionnaire has good test-retest reliability and is stable and credible as a measuring tool for college students' resilience.

This paper examines the structural validity of the scale from two aspects: the first is the correlation degree between different factors and the correlation degree between each factor and the total score. The second is confirmatory factor analysis.

SPSS25.0 software is used to analyze the correlation coefficient, and the correlation between the factors of the scale and the total score of the scale is investigated.  Table 4 is a correlation matrix between factors and total score of college students' resilience scale. It is clearly evident from Table 4 that the correlation coefficient of each factor is between .28 and .62, which is low to moderate positive correlation, and the correlation between each factor is significant (*p* < .01). The correlation between the factors of the scale and the total score ranged from .59 to. 85, which is moderately to highly positive, and all of them are significantly correlated (*p* < .01).

Confirmatory factor analysis is carried out by amoss25.0 software. Taking 26 items obtained from exploratory factor analysis as observation variables, and taking four scale dimensions of “self-efficacy and adaptability,” “negative emotion adjustment ability,” “positive cognition,” and “comprehension and application of social support” as latent variables, a confirmatory structural equation theory model is established.  Figure 1 is correlation matrix between factors and total score of college students' resilience scale. It is clearly evident from Figure 1 that the maximum likelihood method is used in the road map of confirmatory factor analysis.

Table 5 is main model fitting indexes of confirmatory factor analysis. It is clearly evident from Table 5 that the index is less affected by sample size and can properly reflect the fitting degree of the model.

After the path analysis, the factor load of the related items in each dimension of the resilience scale is obtained, and the average variance extraction (AVE) and combined reliability (CR) are calculated.

Table 6 is convergence validity analysis results of resilience scale. It is clearly evident from Table 6 that the factor loads of each topic corresponding to each dimension of the resilience scale are greater than .50, which shows that the topics corresponding to each dimension are highly representative.

The discrimination validity of the scale adopts the method of variance extraction test, that is, if the average variance extraction value of every two dimensions of the scale and the square root of AVE are greater than the correlation coefficient of these two dimensions.

Table 7 is results of discrimination validity analysis of resilience scale. It is clearly evident from Table 7 that there is a significant correlation among the dimensions of the resilience scale (*p* < .01). The absolute value of correlation coefficient of each dimension is less than .50 and less than the square root of the corresponding AVE.

## 5. Conclusion

In this study, Connor-Davidson Resilience Scale is selected as the correlation calibration scale to verify the calibration validity of the self-made college students' resilience scale. 152 college students are selected from Nanjing University of Finance and Economics, and the self-made college students' resilience scale and Chinese version are used to measure the validity of the self-made college students' resilience scale. College students' resilience scale consists of four parts: self-efficacy and adaptability, positive cognition, negative emotion adjustment ability, and comprehension and application of social support. Among them, self-efficacy and adaptability and negative emotion adjustment ability are innovative on the basis of existing research, and understanding the use of social support dimension is the key link between individual internal resources and external resources. College students' resilience scale has good reliability and validity and meets the requirements of psychometrics. It can be used as an effective tool to measure college students' resilience.

## Figures and Tables

**Figure 1:** Confirmatory factor analysis path diagram.

**Table 1:** Factor structure of college students' resilience scale.

Factor	Title number	Load	Common degree
F1	7. I believe in my ability.	.78	.74
	8. I think I can solve the problems I face.	.81	.79
	9. I feel that my existence is meaningful.	.71	.66
	1. I can take care of myself.	.75	.65
	11. When changes happen, I can adapt.	.72	.66
	14. When faced with difficulties, I will make a plan and a solution.	.69	.63
	15. In the face of various pressures, I can adjust or change the original plan in time.	.68	.63
	16. I will come up with a variety of ways to solve the problems I face.	.71	.66

F2	51. I can get emotional support from my family, friends, classmates or teachers.	.77	.72
	52. Someone recognized my worth.	.74	.71
	53. Someone will encourage me.	.79	.77
	54. Someone can really understand me.	.75	.65
	55. Someone can convey positive emotions to me.	.80	.75
	57. When I am caught in a difficult situation in my life, I will take the initiative to seek outside help.	.60	.54
	58. I keep in touch with my family.	.75	.64
	59. When I am upset, I seek comfort and support from my friends.	.73	.63
	62. I can understand other people's feelings.	.58	.53

F3	29. I think the process of things can help people grow more than the result.	.70	.60
	3. I can see the positive side of things.	.62	.68
	31. I will think from a different angle to make myself feel better.	.70	.72
	32. When I encounter difficulties or setbacks, I believe they can give me exercise.	.69	.75
	33. I can look at the problems from multiple angles.	.63	.69

F4	44. I get depressed for no reason.	.73	.60
	45. Unpleasant things bother me for a long time.	.82	.71
	48. I cannot get rid of the memories and fantasies of sad events.	.82	.72
	49. I get caught up in anger and cannot get rid of it.	.82	.71

**Table 2:** Reliability coefficient of internal consistency of college students' resilience scale.

	Stress resistance	Self-efficacy and adaptability	Negative emotion adjustment ability	Positive cognition	Perceive and use social support
*α*	.93	.89	.86	.82	.91

**Table 3:** Test-retest reliability of college students' resilience scale.

	Stress resistance	Self-efficacy and adaptability	Negative emotion adjustment ability	Positive cognition	Perceive and use social support
Test retest reliability	.67	.68	.54	.42	.69

**Table 4:** Correlation matrix between factors and total score of college students' resilience scale.

	Total score of stress resistance	Self-efficacy and adaptability	Negative emotion adjustment ability	Positive cognition	Perceive and use social support
Total score of stress resistance	1				
Self-efficacy and adaptability	.84^∗∗^	1			
Emotional stability	.59^∗∗^	.35^∗∗^	1		
Positive cognition	.78^∗∗^	.62^∗∗^	.28^∗∗^	1	
Social support	.85^∗∗^	.57^∗∗^	.31^∗∗^	.58^∗∗^	1

**Table 5:** Main model fitting indexes of confirmatory factor analysis.

Fitting index	Judgment standard	Results of this study
*CMIN/DF*	<2. When the sample size is large, it can be <5	3.50
*RMSEA*	<.08, preferably <.05	.04
*CFI*	>.90	.97
*NFI*	>.90	.96
*TLI*	>.90	.96

**Table 6:** Convergence validity analysis results of resilience scale.

Dimension	Item	Factor load	Average variance extraction (AVE)	Combination reliability (CR)
Self-efficacy and adaptability	*Q*1	.73	.53	0.9
	*Q*2	.75		
	*Q*3	.79		
	*Q*4	.64		
	*Q*5	.67		
	*Q*6	.72		
	*Q*7	.79		
	*Q*8	.72		

Negative emotion adjustment ability	*Q*9	.73	.62	.87
	*Q*10	.82		
	*Q*11	.85		
	*Q*12	.75		

Positive cognition	*Q*13	.50	.53	.84
	*Q*14	.81		
	*Q*15	.72		
	*Q*16	.78		
	*Q*17	.78		

Perceive and use social support	*Q*26	.58	.54	.91
	*Q*25	.63		
	*Q*24	.62		
	*Q*23	.70		
	*Q*22	.80		
	*Q*21	.77		
	*Q*20	.86		
	*Q*19	.86		
	*Q*18	.75		

**Table 7:** Results of discrimination validity analysis of resilience scale.

	Self-efficacy and adaptability	Negative emotion adjustment ability	Positive cognition	Perceive and use social support
Self-efficacy and adaptability	.53			
Negative emotion adjustment ability	.39^∗∗^	.62		
Positive cognition	.69^∗∗^	.33^∗∗^	.53	
Perceive and use social support	.63^∗∗^	.35^∗∗^	.64^∗∗^	.54
AVE square root	.73	.79	.73	.73

## Data Availability

The simulation experiment data used to support the findings of this study are available from the corresponding author upon request.
